The article "The Application of Knowledge Distillation toward Fine-Grained Segmentation for Three-Vessel View of Fetal Heart Ultrasound Images" was published in 2022. Journal: Comput Intell Neurosci.

# The Application of Knowledge Distillation toward Fine-Grained Segmentation for Three-Vessel View of Fetal Heart Ultrasound Images

**DOI:** 10.1155/2022/1765550

**Published:** 2022-07-14

**Authors:** Qiwen Cai, Ran Chen, Lu Li, Chao Huang, Haisu Pang, Yuanshi Tian, Min Di, Mingxuan Zhang, Mingming Ma, Dexing Kong, Bowen Zhao

**Affiliations:** ^1^School of Mathematical Sciences, Zhejiang University, Hangzhou, China; ^2^Sir Run Run Shaw Hospital, Zhejiang University School of Medicine, Hangzhou, China; ^3^College of Pharmaceutical Sciences, Zhejiang University, Hangzhou, China; ^4^Ningbo First Hospital, Ningbo, China; ^5^The First Affiliated Hospital, Zhejiang University School of Medicine, Hangzhou, China

## Abstract

**Objectives:**

Measuring anatomical parameters in fetal heart ultrasound images is crucial for the diagnosis of congenital heart disease (CHD), which is highly dependent on the clinical experience of the sonographer. To address this challenge, we propose an automated segmentation method using the channel-wise knowledge distillation technique.

**Methods:**

We design a teacher-student architecture to conduct channel-wise knowledge distillation. ROI-based cropped images and full-size images are used for the teacher and student models, respectively. It allows the student model to have both the fine-grained segmentation capability inherited from the teacher model and the ability to handle full-size test images. A total of 1,300 fetal heart ultrasound images of three-vessel view were collected and annotated by experienced doctors for training, validation, and testing.

**Results:**

We use three evaluation protocols to quantitatively evaluate the segmentation accuracy: Intersection over Union (IoU), Pixel Accuracy (PA), and Dice coefficient (Dice). We achieved better results than related methods on all evaluation metrics. In comparison with DeepLabv3+, the proposed method gets more accurate segmentation boundaries and has performance gains of 1.8% on mean IoU (66.8% to 68.6%), 2.2% on mean PA (79.2% to 81.4%), and 1.2% on mean Dice (80.1% to 81.3%).

**Conclusions:**

Our segmentation method could identify the anatomical structure in three-vessel view of fetal heart ultrasound images. Both quantitative and visual analyses show that the proposed method significantly outperforms the related methods in terms of segmentation results.

## 1. Introduction

It is reported that the annual birth rate of congenital heart disease (CHD) in children is 0.8–1% [1, 2], and the incidence rate has ranked first among all birth defects. At present, fetal echocardiography is an important medical imaging technology and most used for prenatal detection and diagnosis of CHD. Well-trained and experienced doctors can make a reliable diagnosis of 80–90% CHD by fetal echocardiography, while the diagnostic accuracy of doctors who lack experience in fetal echocardiography operation and diagnosis is significantly decreased [3, 4].

The three-vessel and trachea (3VT) view is one of the fetal echocardiography views, which was introduced by Yagel et al. [5] as a complementary cardiac view to easily assess the aortic arch anomalies. Gireadă et al. [6] performed a retrospective study on 1,596 unselected pregnant patients presenting at 11–37 weeks of gestation for a routine anomaly scan and analyzed the performance of the four-chamber (4C) view and 3VT view in detecting CHD. The results demonstrated 4C view detected 47.8% of all CHD, going up to 71.7% by adding grayscale 3VT view. The 3VT view is deemed desirable if technically feasible by both International Society of Ultrasound in Obstetrics and Gynecology (ISUOG) and American Institute of Ultrasound in Medicine (AIUM) screening guidelines [7, 8], especially due to its utility in detecting outflow tract anomalies [9–11].

Automatic image segmentation can guide operators to standardize and serialize the display and analysis of fetal echocardiography data. Semantic segmentation has been extensively studied for natural images and is expected to be applied to medical images to assist in diagnosis. However, unlike natural images, medical images are often more difficult to acquire and annotate, which results in a small amount of annotated data. In addition, the special imaging modality (e.g., ultrasound) of medical images produces images of low quality with noises and blurred boundaries. These factors often lead to unsatisfactory segmentation of images. For the segmentation of three-vessel view of fetal heart ultrasound images, we collected a total of 1,300 annotated images, which is completely incomparable to large natural image segmentation datasets.

Recently, machine learning methods have widely used in fetal image processing or ultrasound image processing, such as quality assessment [12–14], detection, and segmentation [15–17]. In the field of vessel image processing, physical models or properties are sometimes introduced to simulate realistic environment to obtain higher evaluation accuracy [18–20].

In this paper, we propose to utilize the channel-wise knowledge distillation [21, 22] technique toward fine-grained segmentation of three vessels in the 3VT view of fetal heart ultrasound images. Particularly, we first train a teacher model whose training data is precisely cropped to a region of three vessels. Such a teacher model enables fine-grained segmentation because it focuses only on the target region. However, such a model cannot be directly applied to the test data because we are not able to crop the test image to the target region before prediction. To this end, we train the student model by distilling the knowledge of the pretrained teacher model using full-size training data. This allows the student model to have both the fine-grained segmentation capability of the teacher model and the ability to handle full-size test images. Experiments show that the proposed method outperforms the most widely used existing methods by a significant margin.

## 2. Methods

### 2.1. Channel-Wise Knowledge Distillation

Knowledge distillation was originally designed for model compression: a compact student model is trained to perform better under the supervision of a large teacher model [23–25]. A subsequent study [26] has also shown that a student model with the same configuration as the teacher model can even exceed the performance of the teacher model. In this work, we employ the channel-wise knowledge distillation method, as it was shown to be more effective than the pixel-wise knowledge distillation that simply aligns point-wise classification scores per pixel [27, 28].

Channel-wise knowledge distillation was first introduced by Zhou et al. [21]. Its basic idea is to convert the feature map on each channel to a probability map and then align the channel-wise probabilities of the teacher model and the student model. The corresponding channel-wise distillation loss ℒ_*C*  *D*_(·, ·) is defined in the form of a KL divergence:

(1) $$\begin{array}{c} {ℒ}_{K\;D}\left(y^{T},y^{S}\right)=\frac{\tau^{2}}{C}\sum_{c=1}^{C}\sum_{i=1}^{W\cdot H}\phi \left(y_{c,i}^{T}\right)\cdot \;\log\left[\frac{\phi \left(y_{c,i}^{T}\right)}{\phi \left(y_{c,i}^{S}\right)}\right], \end{array}$$

where *T* and *S* denote the teacher and student models, *y*^(·)^ denotes the predicted logits of size *H* × *W* × *C*; *i* indexes the spatial location of pixels, where *W* and *H* are the width and height of the predicted logits; *c*=1,2, .., *C* indexes the channel, where *C* is the number of classes including the background; *τ* is a hyperparameter called distillation temperature; *ϕ*(·) is a channel-wise softmax function which converts the logits on each channel into a soft probability distribution, defined as

(2) $$\begin{array}{c} \phi \left(y_{c,i}\right)=\frac{\exp\left(y_{c,i}/\tau \right)}{\sum_{i=1}^{W\cdot H}\exp\left(y_{c,i}/\tau \right)}. \end{array}$$

### 2.2. Our Method

In this paper, we use a model of the DeepLabv3+ [29] architecture with channel-wise knowledge distillation to segment three vessels in 2D fetal heart ultrasound images.

DeepLabv3+ is an encoder-decoder network designed for segmentation tasks. A modified aligned Xception model is used as the encoder, while the Atrous Spatial Pyramid Pooling (ASPP) layer is used as the decoder as the default setting of DeepLabv3+.

As shown in Figure 1, the teacher and student networks use the same architecture. According to the groundtruth label masks, we crop the region of interest (ROI, i.e., the region of three vessels) from full-size images to train the teacher model. Meanwhile, we record the coordinates of cropped regions to restore them to the corresponding spatial location in the full-size image afterwards. After training teacher network with cropped inputs, its logits output is used to distill knowledge on channels for student model training. This allows the student model to have the same ability to segment the ROI as the teacher model. For the training of the student model, we use full-size images as input and align the logits of the teacher model to the full-size ones as additional knowledge. The loss of our network is made up of three components:

(3) $$\begin{array}{c} L=\alpha \cdot {ℒ}_{CE}\left(y_{gt},y_{\text{pred}}\right)+\beta \cdot {ℒ}_{\text{Dice}}\left(y_{gt},y_{\text{pred}}\right)+\gamma \cdot {ℒ}_{K\;D}\left(y^{T},y^{S}\right). \end{array}$$

Here, ℒ_*CE*_(·, ·) and ℒ_Dice_(·, ·) denote cross-entropy loss and dice loss, respectively, *y*_*gt*_ is the groundtruth label mask, and *y*_pred_ is the predicted probability map showing the probability that each pixel being categorized in each class. ℒ_*K*  *D*_(·, ·) is defined in Section 2.1. Note that for the teacher network, *γ* is set to 0, since no knowledge distillation is used.

### 2.3. Materials

1300 pregnant women who underwent fetal echocardiography examination in Sir Run Run Shaw Hospital from 2016 to 2021 were randomly recruited. The gestational age was 20 to 40 weeks. The inclusion criteria were as follows: (1) normal fetus without heart or noncardiac malformations, especially there has no abnormality in the nine standard fetal echocardiography views posted by ISUOG; (2) low risks of chromosome abnormalities were confirmed by early NT and maternal serological examination, or amniocentesis and umbilical cord blood puncture; (3) gestational weeks estimated by ultrasound were consistent with those calculated by menopause history (difference <2 weeks); and (4) the mothers who had no diabetes, hypertension, or pregnancy complications. All pregnant women were informed the purpose of this study and agreed that their fetal heart ultrasound related data should be used for scientific research, and consents should be signed.

Philips IE33 (Philips Medical Systems, Bothell, WA, USA) color ultrasound diagnostic instrument was used, with S5-1 2D imaging probe and a frequency of 1∼6 MHz. Firstly, the fetal echocardiography mode was used to comprehensively evaluate the structure and function of the fetal heart, clearly displaying the standard three-vessel view images and storing the original data. Pregnant women are requested to hold their breath or reduce the range of breathing as much as possible during the whole collection process.

Seven experienced doctors annotated and reviewed the collected fetal heart ultrasound images. They annotated the pulmonary artery (PA), aorta (AO), and superior vena cava (SVC) regions on each image as the groundtruth. The resolution of the original image is 1024 × 768. All images are simply center-cropped and resized to 512 × 512 as full-size training data in the student network. The ROI-based cropped images described in Section 2.2 are generated by padding the annotated three-vessel region with 50 pixels per edge and resizing them to a square region of size 512 × 512. We selected 1040, 130, and 130 images in all experiments for training, validation, and testing, respectively.

Figure 2 shows two examples of the fetal heart ultrasound images, as well as their corresponding full-size labeled images and ROI-based cropped images.

### 2.4. Training

The proposed method is implemented on an NVIDIA RTX 3090 GPU using the Keras and TensorFlow frameworks and trained using the Adam optimizer. We train the network through two stages:

1. During the first stage, the initial learning rate is 0.0005 and the parameters are initialized by pretraining on the PASCAL VOC 2012 [30] dataset. All parameters of the Xception backbone are frozen. We set *α*=1, *β*=1, and *γ*=0. Since the main purpose of this stage is to speed up the training, we do not use the channel-wise knowledge distillation here. The batch size is set to 8.
2. During the second stage, the initial learning rate is 0.00005 and all layers are trainable. We set *α*=1, *β*=1 for both teacher and student models, while the hyperparameters of the channel-wise knowledge distillation are *γ* = 3 and *τ* = 4 and are used only in the student model. In equation (1), *C*=4 as we have 4 classes including the background, PA, AO, and SVC. The batch size is set to 2, since backpropagation to the backbone layers requires a larger amount of GPU memory.

In both stages, we set the decayed learning rate as *lr*=*lr*_init_ · 0.92^iterations−1^ and train for 50 epochs with an early stopping setting when the validation loss stops decreasing.

The following random data augmentation methods are used in the training: scale transformation, displacement, flip, rotation, and color jittering.

## 3. Results

To evaluate the performance of the proposed method, we compare with the most used existing methods, including U-Net [31] and the original DeepLabv3+. U-Net is a classical network and is widely used in medical image segmentation. The original DeepLabv3+ is also adopted as our teacher network; we train it on full-size images for performance comparison. For ablation study, we train the models for comparison by using a combination of cross-entropy loss and dice loss without the knowledge distillation.

To quantitatively evaluate the segmentation accuracy, we use three evaluation protocols: Intersection over Union (IoU), Pixel Accuracy (PA), and Dice coefficient (Dice).

IoU:

(4) $$\begin{array}{c} \text{IoU}=\frac{\left|S_{a}\cap S_{b}\right|}{\left|S_{a}\cup S_{b}\right|}\times 100\%. \end{array}$$

PA:

(5) $$\begin{array}{c} PA=\frac{\left|S_{a}\cap S_{b}\right|}{\left|S_{a}\right|}\times 100\%. \end{array}$$

Dice:

(6) $$\begin{array}{c} \text{Dice}=\frac{2\cdot \left|S_{a}\cap S_{b}\right|}{\left|S_{a}\right|+\left|S_{b}\right|}\times 100\%. \end{array}$$

Here, *S*_*a*_ is the predicted segmentation result of the network and *S*_*b*_ is the groundtruth.

Table 1 shows the performance of our method. We present the IoU, PA, and Dice for each class evaluated on the test data. The mean value over three vessels' segmentation accuracies is shown in the bottom row. The mean IoU, PA, and Dice of the proposed method are 68.6%, 81.4%, and 81.3%, respectively.

Table 2 shows the comparison of three methods. The displayed measurements are the average of the three vessels' segmentation accuracies from all test data. It is evident that the proposed method performs better than the other methods.

To intuitively demonstrate the effectiveness of our results, we plot segmentation contours of the listed methods in Figure 3.

Specifically, we observed that when using existing segmentation methods, the SVC vessel is sometimes undetected or incorrectly segmented due to its small size. In addition, since the three vessels occupy only a small portion of the image, the existing methods only produce rough and incorrectly segmented boundaries.

## 4. Discussion

The incidence of birth defects in China is about 5.6% and the number of new birth defects is about 900,000 every year [1]. Amongst them, there are about 250,000 cases of birth defects that can be observed clinically at birth. Birth defects are the main causes of early abortion, stillbirth, perinatal death, infant death, and congenital disability, which not only seriously harm the survival and quality of life of children but also affect the happiness and harmony of families. It will also lead to potential life loss and increasing social and economic burden. Accurate prenatal diagnosis can significantly improve the perioperative treatment effect of CHD and the success rate of operation and reduce neonatal mortality.

Many studies have shown that improving the ability of routine obstetricians to recognize CHD is the most important issue to improve the successful rate of CHD prenatal diagnosis. However, doctors who complete obstetrical ultrasound diagnoses in their daily medical work are always lacking the diagnostic basis and evaluation experience of complex CHD, and it is difficult to obtain all basic views needed for CHD diagnosis [32–35], including four-chamber cardiac view, left and right ventricular outflow tract view, and three-vessel view, so it is difficult to make reliable display and diagnosis of CHD. As a result, CHD has become the most easily missed structural abnormality in prenatal routine ultrasound examination.

As we know, the 4C view is the most commonly used and easily obtained basic view in fetal heart examination. The acquisition rate at 16–40 weeks is around 95–99.5%, but four-chamber abnormalities only account for 48–63% of congenital cardiovascular malformations. A variety of fetal congenital cardiovascular malformations do not show abnormal shape of the four-chamber heart, including tetralogy of fallot, persistent truncus arteriosus, aortic valve stenosis, pulmonary valve stenosis, transposition of great arteries, and double outlet of ventricle. The extended basic views include three-vessel view, three-vessel trachea view, aortic arch view, pulmonary artery-ductus arteriosus arch view, and vein-atrium connection view. The detection rate of congenital cardiovascular malformation can be increased from 48–63% to 83–86%. Amongst which, the number, internal diameter, course, vascular arrangement, and abnormal blood flow direction of the major vessels can be clearly observed in the three-vessel and three-vessel trachea view, which plays an important role in the screening of fetal cardiac macrovascular malformations. Therefore, it is clinically important to collect and identify the three vessels, and the automatic segmentation algorithm could help doctors to easily operate and accurately diagnose CHD.

Automated segmentation of fetal heart ultrasound images is a challenging task due to low signal-to-noise ratio, low contrast, and blurred boundaries. Collecting and accurately annotating the data is also a difficult task. We believe that the performance of the proposed model can be further improved by using a larger and more standard dataset. Nonetheless, we achieved better results than DeepLabv3+ on all evaluation metrics, with performance gains of 1.8% on mean IoU (66.8% to 68.6%), 2.2% on mean PA (79.2% to 81.4%), and 1.2% on mean Dice (80.1% to 81.3%).

## 5. Conclusion

In summary, we propose a fully automated segmentation method for fine-grained segmentation of three vessels in the 3VT view of fetal heart ultrasound images using a channel-wise knowledge distillation technique. We design a teacher-student architecture to distill channel-wise knowledge from ROI-based cropped images to full-size images. The logits output of the teacher model empowers the student model with fine-grained segmentation capability. In this way, we obtain more accurate segmentation boundaries. Both quantitative and visual analyses show that the proposed method significantly outperforms other methods in terms of segmentation results of the three vessels in the 3VT view of fetal heart ultrasound images.

## Figures and Tables

**Figure 1:** Overview of the proposed channel-wise knowledge distillation method.

**Figure 2:** The 1st column shows original 3VT view of fetal heart ultrasound images. The 2nd column shows full-size labelled images, the red region is pulmonary artery (PA), the green region is aorta (AO), and the yellow region is superior vena cava (SVC). The 3rd column shows ROI-based cropped images, which are cropped from full-size images.

**Figure 3:** Segmentation results of different methods. The original 3VT view of fetal heart ultrasound images are shown in the first column and the groundtruth are shown in the second column. The segmentation results of U-Net, DeepLabv3+ and our proposed method are shown in the last three columns, respectively.

**Table 1:** Performance of the proposed method.

	IoU (%)	PA (%)	Dice (%)
Pulmonary artery (PA)	71.2	83.5	83.2
Aorta (AO)	69.7	82.8	82.1
Superior vena cava (SVC)	64.9	77.8	78.7
Mean	68.6	81.4	81.3

The segmentation accuracies of three vessels and their mean values are shown.

**Table 2:** Performance comparison to existing methods.

	IoU (%)	PA (%)	Dice (%)
U-Net	62.4	77.5	76.9
DeepLabv3+	66.8	79.2	80.1
**Ours**	**68.6**	**81.4**	**81.3**

The mean segmentation accuracy of three vessels over all test data is shown.

## Data Availability

The image data used to support the findings of this study have not been made available due to information that could compromise the privacy of research participants.
